The article "Cyclin H Regulates Lung Cancer Progression as a Carcinoma Inducer" was published in 2021. Journal: Comput Math Methods Med.

# Cyclin H Regulates Lung Cancer Progression as a Carcinoma Inducer

**DOI:** 10.1155/2021/6646077

**Published:** 2021-03-09

**Authors:** Lili Mao, Xu Ling, Ji Chen

**Affiliations:** ^1^Department of Operation Room, Huashan Hospital, Shanghai Medical College, Fudan University, China; ^2^Department of Thoracic Surgery, Huashan Hospital, Shanghai Medical College, Fudan University, China

## Abstract

**Introduction:**

Studies have previously shown that Cyclin H (CCNH) is involved in the tumorigenesis and development of many cancers. The increasing research in CCNH is associated with the poor prognosis of most human cancers. Early diagnosis and clinical treatment are still the main challenges for lung cancer treatment. However, the exact role of CCNH in the tumorigenesis of lung cancer remains unclear.

**Methods:**

The Tumor Genome Atlas (TCGA) database and the Clinical Proteomics Tumor Analysis Association (CPTAC) database were analyzed to detect key genes that might play an important role in lung cancer. The biological functions of CCNH were further revealed through bioinformatics experiments. The Kaplan-Meier method was applied to explore the relationship between CCNH expression and prognosis. Quantitative reverse transcription-polymerase chain reaction (qRT-PCR) was used to detect the expression levels of CCNH in 6 lung cancer tissues and 3 cancer cell lines. The effect of CCNH expression on lung cancer progression was studied by in vitro functional experiments.

**Results:**

Database analysis screened out candidate oncogenes, and CCNH was of great significance to the tumorigenesis of lung cancer. The higher the expression of CCNH was, the lower the survival rate of lung cancer patients were. The qRT-PCR data illustrated that the CCNH expression level was largely increased in lung cancer tissues and cells. The reduction of CCNH inhibited cell proliferation, invasion, and migration.

**Conclusion:**

CCNH was related to poor prognosis, suggesting that CCNH regulated the tumorigenesis and development of lung cancer. Our study suggested that CCNH was a promising biomarker and target in the treatment of lung cancer.

## 1. Introduction

Lung cancer is the primary inducer of cancer mortality worldwide and has changed from a rare disease to a global problem and a public health problem [1]. Patients are usually diagnosed as late-stage because lung cancer does not have obvious changes in early time [2]. In all stages of lung cancer, less than 7% of patients can survive for 10 years after diagnosis [3]. Therefore, early diagnosis and treatment are key factors in reducing mortality and improving patient prognosis. Currently, reasonable use of surgery, chemotherapy, biological targeting, radiotherapy, and other methods is applied to achieve radical cure or maximumly control of tumors, increase the cure rate, improve the quality of life of patients, and prolong life [4]. Ongoing preclinical studies and clinical trials involved in new targeted therapies are expected to ameliorate the survival rate of lung cancer patients [5, 6]. Up to date, the US Food and Drug Administration has approved four targeted therapies for lung cancer treatment: gefitinib (2002), erlotinib (2003), bevacizumab (2006), and crizotinib (2011) [7]. Until now, new medical targets still need exploring for lung cancer treatment.

The article "Cyclin H Regulates Lung Cancer Progression as a Carcinoma Inducer" was published in 2021. Journal: Comput Math Methods Med.

Cyclin H (CCNH) displays importance in carcinogenesis [8, 9]. CCNH is greatly associated with poor clinical-pathological variables in human esophageal squamous cell carcinoma (ESCC) and functions importantly in ESCC tumorigenesis and development. This protein, together with cyclin-dependent kinase 7 (CDK7) and accessory protein MAT1, forms a cyclin activated kinase (CAK) complex [10]. CAK is essential for modulating cell cycle. Wang et al. found CCNH/CDK7 interaction could stabilize C-terminal binding protein 2 and promote cancer cell migration [8]. Besides, CCNH has been found to participate in many cancer progressions. For instance, CCNH is demonstrated to have an association with cell cycle, apoptosis, DNA repair, cell proliferation, and other signaling pathways in breast cancer [11, 12]. The role of CCNH in other cancers also remains to be explored.

Here, TCGA database and CPTAC database were applied to analyze the key genes in lung cancer. We discussed the expression of CCNH in lung cancer and its relationship with clinical parameters. In addition, we carried out biological verification of the function of CCNH in vitro. Thus, we predicted that CCNH might be a promising target therapy for lung cancer.

## 2. Materials and Methods

### 2.1. The Cancer Genome Atlas (TCGA) Database and Clinical Proteomics Tumor Analysis Association (CPTAC) Database

This study analyzed two data sets. The first was TCGA data set, which included RNA sequencing data of all cancer types (http://gdac.broadinstitutewebsite). mRNA expression (raw counts and kilobase transcripts per million (TPM) reads) data were normalized by quantile normalization. The second was the CPTAC data set, which contained the expression level of CCNH protein obtained from the CPTAC (https://cptac-data-portal.georgetown.edu/).

### 2.2. Integration of Protein-Protein Interaction (PPI) Network and Module Analysis

The Interaction Gene Search (STRING) database search tool was applied to validate PPI information. STRING (version 9.0) covered 5214 234 proteins in 1133 organisms. For further evaluating the interplay between the differential expression, we mapped the differential expression to STRING, and only the comprehensive score verified by experiments was significant. Then Cytoscape software was applied to construct the PPI network. The cytokeratin (PPI) network module was screened using plug-in molecular complex detection (MCODE) technology. The standards were listed as follows: MCODE scores and the number of nodes. *P* < 0.05 was considered a significant difference.

The article "Cyclin H Regulates Lung Cancer Progression as a Carcinoma Inducer" was published in 2021. Journal: Comput Math Methods Med.

### 2.3. Clinical Specimens

Clinical tissues from lung cancer and normal tissues from six patients who obtained informed consent were tested and compared here. All lung cancer patients were treated in Huashan Hospital. The samples of lung cancers patient were confirmed histopathologically and kept at -80°C for the following use. Our study and experimental procedure were approved by the hospital's Human Subjects Committee.

### 2.4. Cell Culture and Transfection

Human normal lung cell lines (MRC-5) and human lung cancer cell lines (H1299, A549 and Calu-1) were obtained from the Cell Bank of Type Culture Collection (CBTCC, Chinese Academy of Sciences, Shanghai, China). All cells were maintained in DMEM (Gibco, Carlsbad, CA) with 10% FBS (BI, Israel) under 37°C incubators with 5% CO_2_.

When the cells reached 70% confluence, the cells used for transfection were plated in a 6-well plate. CCNH knockdown was done using two different designed siRNAs (Cyagen, Guangzhou, China). siRNAs were transfected into A549 and H1299 cells using Lipofectamine 3000 (Invitrogen, Carlsbad, CA). After 6 hours, the fresh medium was changed and cells were cultivated for another 24 hours. The siRNA sequence was used in the experiment as follows: si-CCNH-1, 5′-CCTGCAAAGTAGATGAATTTT-3′; si-CCNH-2, 5′-CCACCTTATTGTCCACAATTT-3′; and si-NC, 5′-UUCUCCGAACGUGUCACGUTT-3′.

### 2.5. RNA Isolation, cDNA Synthesis, and Quantitative Real-Time PCR

Trizol solution (Invitrogen, USA) was applied to extract the whole RNA from cells or tissues. PrimeScript RT kit and SYBR Premix Ex Taq (Vazyme, Nanjing, China) were conducted to perform qRT-PCT analysis as the manufacturer's instructions. Our results were normalized to the expression of glyceraldehyde-3-phosphate dehydrogenase (GAPDH). qRT-PCR results got analyzed to obtain the Ct value of the amplified product, and the data were analyzed by the 2^-*ΔΔ*Ct^ method. Specific primers used were as follows: CCNH—forward: 5′-TGTTCGGTGTTTAAGCCAGCA-3′, reverse: 5′-TCCTGGGGTGATATTCCATTACT-3′; GAPDH—forward: 5′-GGAGCGAGATCCCTCCAAAAT-3′, reverse: 5′-GGCTGTTGTCATACTTCTCATGG-3′.

### 2.6. Cell Proliferation Assay

Cell proliferation was assessed by cell counting kit 8 (CCK-8) (Dojindo, Japan). Si-CCNH-transfected A549 and H1299 cells were reseeded on 96-well plates as indicated. 10 *μ*L of CCK-8 was added to per well at 0 h, 24 h, 48 h, 72 h, and 96 h time points and maintained for 2 hours. The absorbance value (OD) of 450 nm was measured on a microplate reader.

The article "Cyclin H Regulates Lung Cancer Progression as a Carcinoma Inducer" was published in 2021. Journal: Comput Math Methods Med.

### 2.7. Transwell Assay

The Transwell chamber (pore size 8 *μ*m, Corning) was used for cell migration and invasion assays. The Transwell chamber was coated with Matrigel, and 500 *μ*L medium supplied with 20% FBS was added into the lower chamber. 200 *μ*L medium absence of serum containing 6 × 10^4^ H1299 cells was added into the upper chamber. After 20 hours, the cells were fixed in formaldehyde for 10 minutes and stained with DAPI. After 20 minutes, the sample was washed, dried, and fixed on a glass slide. The migrating cells that were stained blue were observed under an inverted microscope, and five areas were randomly selected for statistics.

### 2.8. Statistical Analysis

SPSS 17.0 software was applied to analyze the data. Student's *t*-test was conducted to analyze the differences between groups. One-way ANOVA was conducted to compare multiple groups. The survival probability was analyzed by the Kaplan Meier method and calculated by the log-rank test. ^∗^*P* < 0.05, ^∗∗^*P* < 0.01, and ^∗∗∗^*P* < 0.001 indicated significant difference.

## 3. Results

### 3.1. PPI Networks of Lung Adenocarcinoma (LUAD)

The PPI network of LUAD's differential expressed genes (DEGs) was composed of 70 nodes and 29 edges (Figure 1). Given the string database information, the top nodes with higher node degrees were selected. These gene centers included cyclin H (CCNH), lipolysis-stimulated lipoprotein receptor (LSR), retinal outer segment membrane protein 1 (ROM1), phosphatidylinositol glycan anchor biosynthesis class C (PIGC), and pure nucleoside phosphorylase (PNP). CCNH possessed the highest node degree amid all selected genes.

### 3.2. The Clinical Significance of CCNH Protein Expression Level

Based on the bioinformatics analysis of the CPTAC database, we constructed the relationship between the level of CCNH protein expression and the grade, gender, age, weight, and tumor stage of LUAD patients. Our data showed that the CCNH protein expression level of LUAD patients was positively correlated with tumor grade (Figure 2(a)), and the increase in CCNH protein expression level was positively correlated with the patient's gender (Figure 2(b)). However, the correlation between CCNH expression and tumor grade and the correlation between gender differences in LUAD patients had not been found yet. The expression level of CCNH protein was positively correlated with the age of LUAD patients (Figure 2(c)) but negatively correlated with body weight. However, the difference in CCNH protein expression in obese patients was minor (Figure 2(d)). In addition, we found that the levels of CCNH protein in various cancers were different (Figure 2(e)), and the level of CCNH protein expression in each stage of LUAD was higher than normal (Figure 2(f)).

The article "Cyclin H Regulates Lung Cancer Progression as a Carcinoma Inducer" was published in 2021. Journal: Comput Math Methods Med.

### 3.3. CCNH Was Related to Lung Cancer Progression and Differentially Expressed in Lung Cancer Tissues and Cell Lines

We conducted Kaplan-Meier method analysis (log-rank test) on TCGA database to explore the association between CCNH expression and prognosis in lung cancer. We observed that the high expression of CCNH was significantly associated with shorter disease-free survival both in patients with LUAD and Lung squamous cell carcinoma (LUSC) (Figures 3(a) and 3(b)). Also, we found that overexpression of CCNH was associated with worse first progression in lung cancer samples (Figure 3(c)). In this study, we also detected the level of CCNH in lung cancer tissues.  Figure 4(a) illustrates that the CCNH expression level in lung cancer tissues was largely higher, compared to that in normal controls. We also got similar results in CCNH cell lines (Figure 4(b)).

### 3.4. CCNH Induced Lung Cancer Cell Proliferation

We further detected the effect of CCNH on cell growth upon ablating CCNH in A549 and H1299 cells. In this study, we designed 2 siRNAs to knock down CCNH. Through qRT-PCR, we found that the knockdown efficiency of siRNA-CCNH-2 was too low (data are not shown), so we chose siRNA-CCNH-1 to knock down CCNH (Figures 5(a) and 5(c)). CCK-8 assay data showed that si-CCNH-transfected A549 and H1299 cell proliferation was reduced when compared with empty vector-transfected cells (Figures 5(b) and 5(d)). It could be inferred that CCNH had a positive relation with cell proliferation.

### 3.5. CCNH Induced Lung Cancer Cell Invasion and Migration

At last, we validated the influence of reduced CCNH on cell invasion and migration. H1299 cells were chosen for studies because of knockdown efficacy. H1299 cells transfected with siRNA targeting CCNH showed that cell migration and invasion were obviously inhibited (Figure 6). CCNH might play an oncogenic role in lung cancer progression.

## 4. Discussion

Nowadays, lung cancer has become a global issue concerning human health. The study of lung cancer never stops [13]. So far, a lot of achievements, including the aspects of lncRNA and circRNA, have been made in lung cancer research. For example, Loewen et al. discussed the functions of lncRNA HOTAIR in lung cancer [14]. Li et al. thought circular RNAs were important molecular modulators and prospective biomarkers for diagnosis and prognosis of non-small cell lung cancer [15]. As for mRNAs, they usually function as the downstream targets [16]. Their roles in lung cancer stay to be discussed.

The article "Cyclin H Regulates Lung Cancer Progression as a Carcinoma Inducer" was published in 2021. Journal: Comput Math Methods Med.

A PPI network with DEGs was established, and the top degree hub genes were listed: CCNH, LSR, ROM1, PIGC, and PNP. Among these genes, CCNH had the highest value. As a member of the cyclin family, Cyclin H forms the CDK-activating kinase (CAK) trimeric complex together with CDK7 and MAT1, which is pivotal for cell cycle and viability modulation [17, 18]. Aberrant expression of cyclin H is shown in multiple tumors, including breast cancer [19], esophageal cancer, endometrial cancer [20], and gastrointestinal stromal tumors [21]. Nevertheless, the clinical significance and biological function of cyclin H in lung cancer are yet elusive.

The development of tumors is a complex process driven by specific genetic and epigenetic changes [22]. In serous ovarian cancer, the researchers verified the relationship between the modules of gene expression and the stage or grade of tumor in five independent data sets [23]. Our data revealed that the CCHN expression level had a certain correlation with tumor stage or grade. This result probably made development into a more objective scoring system, thus improving the forecaster of LUAD results. Alzheimer's disease (AD) is an age and gender-related brain disease [24]. In multiple sclerosis (MS), women are found to have a higher risk of disease than men, and aging-related diseases show obvious gender bias [25]. Here, the CCHN expression level displayed a positive correlation with the age not the gender of LUAD patients. Obesity was reported to be associated with increased cancer incidence and progression in various types of tumor [26]. Obesity is also a central risk factor for many cancers, particularly breast cancer. Breast cancer patients who are overweight or obese or have a disease history perhaps increase the risks of morbidity, recurrence, and breast cancer-related mortality [27]. Obesity is probably bad for life quality, usually generating sexual dysfunction, neuropathy, cardiotoxicity, chronic fatigue, and lymphedema [28]. Our results displayed that the CCHN expression level had a positive correlation with the weight of LUAD patients, but not with obese patients. Additionally, our data demonstrate that CCNH expression levels in different cancers are quite different, and CCNH probably becomes a biomarker for cancer identification.

Clinical studies have demonstrated that there is an association among tumor stage, grade and clinical prognosis [29]. Identifying promising clusters of coexpressed genes of representative stages or grades-associated biomarkers might be conducive to revealing the mechanisms of the tumorigenesis and development of a tumor and predicting patient prognostication. TCGA data sets were applied to study the association between CCNH expression and poor prognosis in LUAD patients. Here, our study tried to study the mode of action of CCNH in lung cancer patients. Our data revealed that lung cancer highly expressed CCNH. Highly expressed CCNH promoted cancer cell viability. Our study displayed that CCNH might display as an oncogene in lung cancer and induce its tumor viability, invasion, and migration.

The article "Cyclin H Regulates Lung Cancer Progression as a Carcinoma Inducer" was published in 2021. Journal: Comput Math Methods Med.

This study has some limitations. It is necessary to detect the expression level of CCNH in more clinical samples. In future studies, we will collect more clinical samples to explore CCNH mRNA and protein expression levels, as well as the correlation between CCNH expression and clinical parameters (including clinical stage, age, and survival time). Besides, we will conduct *in vivo* experiments to further explore the role of CCNH in lung cancer.

To sum up, we validated CCNH expression and function in lung cancer progression through bioinformatics analysis and functional assays for the first time. Through the PPI network, we have identified genes that might play a key role in lung cancer. Based on database analysis. We analyzed the correlation between CCNH and the clinical characteristics of lung cancer patients. CCNH was an important indicator of poor prognosis for lung cancer patients. Our data revealed that CCNH highly expressed in lung cancer cell lines and tissues. Reduced CCNH could inhibit lung cancer cell growth, migration, and invasion. Perhaps, CCNH becomes one of the most valuable prognostic and therapeutic biomarkers of lung cancer. We hope the findings could facilitate lung cancer treatment.

## Figures and Tables

**Figure 1:** The protein-protein interaction (PPI) network of potential protein-related complexes in LUAD.

**Figure 2:** (a) The relationship between the expression of CCNH protein and the grade of LUAD in the CPTAC database. (b) The relationship between the expression of CCNH protein and the gender of LUAD patients in the CPTAC database. (c) The relationship between the expression of CCNH protein and the age of LUAD patients in the CPTAC database. (d) The relationship between the expression of CCNH protein and the weight of LUAD patients in the CPTAC database. (e) The expression level of CCNH protein in various cancers in the CPTAC database. (f) The relationship between the expression of CCNH protein and the tumor stage of LUAD patients in the CPTAC database. The *x*-axis represents the grade/gender/age/weight/tumor stage of LUAD patients or other cancers, and the *y*-axis represents standard deviations from the median across samples for the given cancer type. Log2 spectral count ratio values from CPTAC were first normalized within each sample profile, then normalized across samples.

The article "Cyclin H Regulates Lung Cancer Progression as a Carcinoma Inducer" was published in 2021. Journal: Comput Math Methods Med.

**Figure 3:** (a, b) The Kaplan-Meier method was used to analyze the expression level of CCNH and disease-free survival in patients with LUAD or LUSC. (c) The Kaplan-Meier method was used to analyze the expression level of CCNH and first progression in patients with lung cancer.

**Figure 4:** (a) The expression level of CCNH in tumor tissues and normal tissues. (b) The expression of CCNH in lung cancer cell lines and normal cells. ^∗^*P* < 0.05 and ^∗∗^*P* < 0.01.

**Figure 5:** (a, c) siRNA was used to knock down the level of CCNH in lung cancer cells A549 and H1299. (b, d) CCK-8 was employed to detect the effect of si-CCNH on the proliferation of lung cancer cells A549 and H1299. ^∗^*P* < 0.05.

**Figure 6:** (a, b) The effect of si-CCNH on cell invasion and migration was detected in H1299 cells. ^∗^*P* < 0.05.

## Data Availability

The data that support the findings of this study are available with approval from the author.
